RETRACTED

# Research on Four-Dimensional Innovative Intelligent Education Platform Based on Cloud Edge-End Architecture

**DOI:** 10.1155/2023/2263033

**Published:** 2023-03-01

**Authors:** Buyu Wang, Jingwei Qi, Xiaoping An, Jiangyin Fu, Yuan Wang, Na Liu, Meian Li

**Affiliations:** ^1^College of Computer and Information Engineering, Inner Mongolia Agricultural University, Hohhot 010018, Inner Mongolia, China; ^2^Key Laboratory of Smart Animal Husbandry, Universities of Inner Mongolia Automomous Region, Hohhot 010018, Inner Mongolia, China; ^3^College of Animal Science, Inner Mongolia Agricultural University, Hohhot 010018, Inner Mongolia, China; ^4^Department of Electrical and Computer Engineering, Tandon School of Engineering, New York University, New York, NY 11201, USA

## Abstract

In order to solve the problem of backward talent training mode in agriculture-related colleges and universities, this paper proposed a scheme to build a smart teaching platform by using cloud architecture, combining virtualization and twinning technology. The intelligent teaching platform is developed using the 5G converged network architecture and cloud edge system architecture. The intelligent teaching platform has realized such teaching modes as real scene teaching, combination of virtual and real teaching, immersive teaching, multi-teacher collaborative teaching and live interactive teaching. The smart teaching platform has established a new model of digital education, with the functions of teaching, teaching research, teaching management and teaching evaluation, and provides smart teaching cloud services for teachers and students of agriculture-related colleges and universities as well as external tutors. The research of multi-dimensional evaluation system solves the precise management of teaching process. The teaching effect has been significantly improved, and the management cost has been reduced, which meets the goal of training new agricultural talents in agricultural and forestry colleges.

## 1. Introduction

How to cultivate applied talents required by the development of global agriculture 4.0, how to achieve accurate evaluation of education quality, and then realize the implementation of new agricultural science construction, are the core issues of intelligent education research in animal husbandry discipline.

Cai et al. [1] do to wisdom education curriculum design of exploratory research, puts forward adopting the micro-course or animation display before the class, for students in the class group autonomous teaching and carry out online teaching practice after class in the method of combining effectively promote the students' autonomous learning ability and innovation ability, which laid a foundation for further enhance the level of talent training. Tai et al. [2] pointed out that the reconstruction of smart teaching environment is the deep integration of information technology and education and teaching, which is a higher form of education informatization. He studied the construction of smart teaching environment and proposed the environment construction standard of “interconnection, accurate service and data support”. Gu and Zhang [3] pointed out that wisdom space by classroom teaching equipment management, teaching management, students' attendance management and remote interactive teaching management software and hardware space composition, and the wisdom of teaching space modeling were studied, based on the cloud-side together the wisdom of the education system, solved the “full content and full time domain, the whole process, all terminal, the whole audience” teaching management needs, Fill the gap in the industry. Xu et al. [4] conducted in-depth research on the intelligent teaching system based on artificial intelligence (AI) and computer technology, and found that the application of the intelligent system not only helped students improve their learning efficiency by 9.8%, but also was favored by 56.8% of teachers and students. Gao's [5] research for conducting scientific and objective of education quality evaluation conducted in-depth research, use of big data and artificial intelligence technology to build a quantitative evaluation index system of university teachers' teaching quality and quantitative methods of research and the realization method of intelligent as well as the construction of university teachers' teaching quality quantitative evaluation system of research and implementation method, The authors explores the technical way to find the effectiveness of measurable factors in the evaluation of teaching quality, and the results have important practical significance for scientific evaluation of teaching quality. Zeng's [6] research has applied virtual reality (VR) technology to the intelligent multimedia remote teaching system, and used VR technology to complete the reasonable allocation of multimedia teaching resources and effectively improve the quality of multimedia teaching. Intelligent multimedia distance teaching system can effectively reduce the transmission energy and signal to noise ratio of teaching resource data, which has certain practical value.

RETRACTED

The training of compound applied talents in colleges and universities mainly includes skill type and applied research type. The skilled, represented by higher vocational colleges, have conducted extensive research and exploration on the skilled intelligent education. The most representative is Yu's [7] proposal of how to better cultivate the intelligent teaching model of global industry 4.0 talents under the background of 5G, which connects the four educational links of “teaching, learning, evaluation and capital”. The exponential intelligent teaching mode should be implemented from the aspects of teaching methods, learning forms, evaluation systems and teaching resources. However, there are also some problems such as low enthusiasm of teachers to carry out smart teaching, single smart teaching model and serious fragmentation of resources. For undergraduate education, intelligent education focuses on the application of the cultivation of research talents, Yuan and Li [8] from policy management perspective, put forward the “management, professorial teaching, environment, resources, training objectives,” five elements of M-PERT model, for the building of the model and its effectiveness done in-depth research, verified the value of intelligent education. Intelligent education in colleges and universities not only covers environmental construction, software and hardware support, but also analyzes the application potential and technical application level of intelligent objects in combination with educational theory and practice, and constructs practical application scenarios for different application objects, in application fields, and implementation paths for more application fields. Promote the cloud, intelligent, virtual, two-way evaluation of education services, solve the openness, diversity, collaboration, fairness and sustainability of education, build an intelligent teaching platform, and realize the revolutionary reform of education [9–14].

To sum up, a lot of research work has been done on the use of Internet of Things technology and artificial intelligence technology to carry out intelligent education, and a series of research results have been obtained from teaching activities, teaching management, curriculums construction to teaching evaluation. However, there are two problems: first, all the research focuses on the field of engineering education, and there is no relevant research on the wisdom education of animal husbandry. Secondly, all the studies did not propose how to build a unified cloud platform to carry out intelligent education in the whole process of education. Aiming at the goal of talent training in animal husbandry in agricultural universities in the future, the intelligent education platform composed of 5G converged network [15, 16], intelligent teaching data center, intelligent teaching resource sharing and intelligent teaching cloud service system is researched and constructed by using advanced intelligent technologies such as Internet of Things, cloud computing, big data, artificial intelligence and virtual reality. A linkage closed-loop talent training mode with four dimensions(teaching, teaching research, teaching management and teaching evaluation) of mutual empowerment has been constructed, put forward the four dimensions(multimedia teaching, the teaching of actual scenario and combination of virtual and real teaching and wisdom breeding double team teaching) of teaching mode, solve the problem of the new agricultural livestock disciplines personnel training, The intelligent teaching cloud platform including teaching, teaching research, teaching management and teaching evaluation has been established.

RETRACTED

The contribution of this paper mainly has four aspects. Firstly, the architecture and functional architecture of intelligent teaching cloud platform based on cloud edge and end collaboration are proposed. Secondly, the integrated network architecture based on 5G is proposed to reconstruct the teaching space management, which provides support for the development of intelligent teaching management and accurate teaching evaluation. Third, new teaching resources for animal husbandry have been established, including real scene resources of livestock farms, virtual reality resources and smart breeding digital resources. Fourth, the cloud service system of teaching, teaching research, teaching management and teaching evaluation is studied, which makes exploration and research for the establishment of a universal cloud platform of intelligent education for animal husbandry discipline.

## 2. Intelligent Education Platform Architecture

The architecture of the intelligent education platform adopts cloud edge architecture, and the application architecture adopts multi-level application architecture with security and standards as two wings, as shown in Figure 1. The standard wing mainly includes teaching standards, resource standards, terminal access standards, breeding business standards and livestock data standards. The safety wing mainly includes biological safety, production safety and food safety. The multi-layer application consists of the basic software and hardware platform layer, data resource layer, education service support layer, intelligent education application system layer, and user layer. The basic platform layer is the system hardware and software platform needed to support the system operation. The data resource layer contains all the underlying databases of the platform. Business support layer is the middleware necessary to support system operation. The application system layer embodies the function of intelligent teaching cloud service, which consists of teaching, teaching research, teaching management and teaching evaluation. The platform provides intelligent education services for teachers and students of agricultural and forestry universities, off-campus tutors, teaching administrators and platform operation and maintenance personnel.

RETRACTED

As can be seen from Figure 1, the cloud platform is a five-layer application architecture with security and standards as its two wings. The five layers include foundation layer, data layer, business layer, application layer and user layer. The foundation layer consists of system software, system hardware and data acquisition and rendering system. The system software includes three sets of Smart Teaching Cloud Management System, Operating System and Database Management System. The system hardware includes Cloud Hardware System, Breeding Data Acquisition Terminal, Intelligent Washing Terminal System, and Basic Wireless Network Support System and LABS Share Hardware System five sets of hardware systems. The data acquisition and rendering system consists of Real Scene Data acquisition System, Virtual Simulation Display System, and Virtual Simulation Creation System, Teaching Hardware System and AI Visual Analysis System five sets of hardware and software integrated data acquisition and rendering systems. The hardware system provides hardware computing, storage and network services, the system software provides node operating system, cloud management system and database level system management functions, and the data collection and rendering system provides services for platform data collection, processing, rendering and display. The data layer consists of Breeding Real Scene, Breeding Environment, Individual Sign Database, VR Model Database, and Individual Recognition Training Set, Animal behavior recognition, Individual Identification and other 13 structured and unstructured databases. The business layer consists of the Intelligent Teaching Data Center Platform and the Intelligent Teaching Resource Sharing Platform. The teaching business support layer provides data distribution and sharing services for the data layer and application layer. The application layer consists of Intelligent Teaching Creation System, Intelligent Teaching and Research System, and Intelligent Education Management System, Intelligent Evaluation System, Carrier Open Sharing System, Intelligent Open Classroom Teaching Subsystem, Multi-Division Cooperative Teaching Subsystem, Immersive Presentation System, Intelligent Teaching Subsystem, Four Dimensional Wisdom Teaching System is composed of 10 systems, providing users with a full range of intelligent teaching services from teaching, teaching research, teaching management to teaching evaluation. The user layer consists of college students, college teachers, outside experts, business mentors, and teaching managers, and provides services for the above five types of users.

RETRACTED

Aiming at the privacy and security protection of multi-terminal data in cloud edge architecture, in-depth research is carried out from three aspects: formal verification of security, analysis of attack mechanism and construction of defense strategy. The data processing model of data layer is verified by security formalization, and the complex data processing model which is difficult to explain is transformed into a clearer form of logical constraints. Interpretable adversarial attack generation mechanism analysis method and high-dimensional feature space geometry analysis, decision transfer pathway detection, feature information attribution and visualization techniques are used to analyze the attack generation mechanism to ensure data security.

## 3. Network Architecture of Intelligent Education Platform

The network architecture of the intelligent teaching platform adopts the cloud side-end collaborative network architecture, and the edge and access mobile network adopt 5G converged network [17]. The backbone network mainly consists of the server corresponding to the platform, network and communication system, storage and backup system, network security system, data forwarding system and edge fusion network system. The converged network architecture is shown in Figure 2.

As can be seen from FIG.  2, the 5G converged network is composed of the Internet of Things acquisition terminal network, edge computing network, data center network and network security system. It provides the cloud platform with the fusion network architecture of cloud edge and end cooperation, ensures the network is stable and reliable, and the commercial privacy of data collection is effectively protected. The farm consists of poultry farms (laying hens, etc.) and livestock farms (horses, cattle, sheep, pigs, etc.). The network of IOT collection terminals in breeding farms is composed of four dimensions: Environment Sensor (5 Para), Cameras, individual signs, and handheld Terminals. The edge network uses 5G mobile standby network and WIFI wireless coverage working network to achieve full coverage, with bandwidth ranging from 20 Mbps to 100 Mbps. The data center network consists of Big Data Research, Business Cloud Services, Smart Education Data Center, and Smart Education Resource Sharing Center consists of four service data centers, which provide network support for data management, scientific research, data sharing and cloud services. The internal core exchange loan is 10 Gbps. It provides security systems ranging from firewall, fortress machine and online behavior management. The commercial data is calculated on the edge server, and the desensitized data is stored in the cloud data center, which ensures the commercial privacy security of the farm data.

RETRACTED

The cloud edge-end architecture is an integrated 5G fusion network with low delay, high speed and large capacity from cloud (intelligent teaching data center), edge (edge computing network and edge computing node of school-enterprise cooperation base) to end (sensing terminal, 5G handheld terminal, 5G mobile terminal and various VR/AR terminals). Implement equipment, network infrastructure at the level of unity can be run through the cloud platform promotion goal, completely solve high network latency, low bandwidth, network, the problem of abort, frequently for subsequent development from the teaching, research, teaching research to the evaluation of low latency and high bandwidth, high availability, regulation of 5 g converged network service support.

## 4. Research of Intelligent Teaching Data Center System

The intelligent teaching data center system provides computing, storage, data services and basic business support for the intelligent teaching platform. It is composed of cloud pipe system, cloud real big data management, data processing, data integration and asset management subsystems. Build a 5G fusion network based on 5G technology and cloud side-end architecture, collect four-dimensional cloud panoramic data, establish real data assets, achieve the construction of four-dimensional real scene to simulation panorama of environment (5 Parameters are temperature, humidity, carbon dioxide, ammonia, hydrogen sulfide), scene, process and physical signs, and realize the collection, fusion, storage and asset services of four-dimensional real scene/panoramic data. The system adopts a three-layer architecture to carry the business, namely, the cloud layer, the basic cloud platform and the cloud service. Among them, the cloud layer mainly includes the data sensing end, acquisition terminal, edge computing terminal, data forwarding node, 5G terminal and standby 5G network to complete data collection and primary filtering functions. The basic cloud platform mainly includes cloud storage, cloud computing, and 5G cloud switching. Cloud services mainly include cloud teaching, cloud teaching research, cloud teaching management and cloud teaching evaluation services.

Wisdom teaching data center system, provide for industry application in the field of teaching immersive anytime and anywhere in the wisdom of open classroom (cloud online courses, more open, collaboration in interactive teaching in classroom and wisdom open class), live interactive teaching (panoramic live interactive teaching, the four-dimensional live interactive teaching, wisdom, open class) and the actual situation combined with teaching practice. The system architecture of intelligent teaching data center is shown in Figure 3.

RETRACTED

As can be seen from Figure 3, the architecture of Intelligent Teaching Data Center System is a typical cloud edge architecture, consisting of three layers: Edge of Cloud Terminal, Cloud Platform and Cloud Service. Edge of Cloud Terminal mainly completes the collection of real environment data, scene data, process data and individual physical signs data. The Cloud Platform mainly completes the computation, storage, fusion and sharing tasks of structured, semi-structured and unstructured data. The Cloud Service provides teaching, teaching research, Teaching management, and teaching evaluation services for users.

In order to solve the problem of real-time and anywhere immersive teaching in the practice base, real scene collection, construction of immersive virtual simulation resources and cloud distribution to the data center, to provide support for the development of real scene/panoramic online teaching. Through digital twinning technology, the production process twinning of the practice base is built into teaching resources to provide real production process support for intelligent teaching. The collection of the environment of the practice base and the real scene of the individual physical signs of the practice object realizes the overall digital materialization learning from the group to the individual. Based on the cloud-side 5G fusion network, real-time collection and fusion of the 4d real scene of the practice base are realized to generate real-time data assets, providing basic real-time panoramic data support for further realizing real-time control of production process, real-time access of teaching process and real-time analysis of scientific research process.

## 5. Research of Intelligent Teaching Resource Sharing System

The intelligent teaching and training resource sharing platform, relying on the cloud animal husbandry resource sharing platform and using 5G edge network, can meet the needs of users to access the platform anytime and anywhere to obtain shared resources, and provide the resource support required for the “5G + Cloud animal husbandry” intelligent teaching and training platform. The platform consists of data resource sharing system, teaching resource sharing system, platform resource sharing system and carrier resource sharing system., respectively, to provide users with data from the assets (wisdom breeding four-dimensional imaging data, breeding the four-dimensional imaging fusion breeding four-dimensional imaging teaching material data resources, virtual simulation model, individual animals recognition training set data, animal contour recognition training set data, animal behavior recognition intensive track training set data), teaching resources, animal husbandry and teaching resources, Virtual simulation of teaching resources and teaching resources, combining false and true collaboration in twin teaching resources, teaching resources, digital teaching resources of the VR/AR), the platform resources (intelligence cultivation platform resource sharing systems, visualization analysis of environmental data sharing system, the big development suite sharing system, animal behavior analysis system, cloud recognition system, cloud, cloud collaboration system diagnosis and treatment, live teaching system Training system), carrier resources (intelligent teaching virtual simulation creation carrier resources, intelligent teaching digital twin creation carrier resources, intelligent teaching collaborative creation carrier resources, intelligent teaching immersive display carrier resources, AI visual analysis carrier resources, cloud desktop carrier resources).

RETRACTED

As can be seen from Figure 4, the Intelligent Teaching Resource Sharing System provides four types of sharing services: data Resource Sharing, Teaching Resource Sharing, platform Resource Sharing, and carrier Resource Sharing. Data resource sharing provides multi-tenant sharing, API data sharing, and swap space sharing. Teaching resource sharing mainly consists of real scene material sharing, virtual reality teaching resource sharing and animal husbandry course resource sharing. Platform resource sharing mainly includes big data analysis platform and visual big data analysis platform for animal husbandry professional users. Carrier resource sharing is composed of virtual simulation carrier resource sharing, digital twin carrier resource sharing, remote collaboration carrier resource sharing, virtual and real carrier resource sharing, cloud desktop carrier resource sharing. Through the sharing mechanism of the above four kinds of resources, the all-round sharing of teaching resources is realized and the sharing support for the intelligent education cloud platform is provided.

The system provides different recommender services for different users. The system can record users' multi-dimensional cognitive information [18], such as resource discipline, quantity, frequency, comments, likes, forwarding, expressions, to provide support for users to make complex sharing decisions and recommendations in the big data environment. In view of user preference fuzzy probability [19], a Bernoulli matrix decomposition recommendation algorithm based on intuitionistic fuzzy set is used to recommend shared resources for target users [20]. Three-layer Agent is designed to implement intelligent resource sharing recommendation. Agent 1: With the help of the relevant theoretical knowledge of intuitive fuzzy set, the user preference rating matrix is transformed into membership matrix, non-membership matrix and hesitation matrix; Agent 2: Use Bernoulli matrix decomposition model to fit 0–1 matrix in parallel to get the best set of potential feature vectors; Agent 3: The inner product of the feature vector of the matrix is divided and sorted proportionally to determine the intuitionistic fuzzy number favored by the target user. According to the comparison rules of intuitionistic fuzzy number, the intuitionistic fuzzy number set of the resources applied by the user is resorted, and the top one is selected as the recommended application resources.

RETRACTED

## 6. Research of Intelligent Education Cloud Service System

Relying on the intelligent teaching data center and resource sharing center system, the construction of intelligent teaching cloud service system serves the construction of first-class specialty, promotes intelligent education and realizes the subversive revolution of teaching. Through the combination of virtual simulation and real scene panorama, traditional classroom, smart classroom, innovative practice and smart teaching are combined to open up new teaching approaches and realize new teaching forms. The intelligent teaching cloud service system is composed of four systems: intelligent teaching subsystem, intelligent teaching and research subsystem, intelligent teaching tube system and intelligent teaching evaluation subsystem. It provides users with real-scene teaching, virtual simulation teaching, immersive role-playing practice teaching, live interactive teaching and panoramic interactive live teaching. Carried out from the open classroom wisdom (cloud online courses, more open classroom, multi-dimensional holographic wisdom and open teaching, open hole 3 d class), teaching and research of cloud (cloud evaluation, immersive panorama online tour lecture), cloud taught tube (5 d open classroom/laboratory, equipment intelligent inspection) to the intelligent evaluation (teaching process evaluation, study effect evaluation) of disruptive innovation.

### 6.1. Research of Intelligent Teaching Subsystem

The intelligent teaching subsystem mainly carries out four-dimensional teaching composed of four dimensions: traditional multimedia, real scene panorama, virtual simulation and industry intelligent production. Based on cloud architecture of fusion network, the design of the open classroom, four-dimensional bricks, many live together and trainers, and other functions module, give full play to the 5 g low latency, high rate and large capacity, the characteristics of the integrated use of based on artificial intelligence, big data, cloud computing, Internet of things, virtual simulation, such as information technology, around the “teaching and research, tubes, review” and other key areas of teaching link, It provides convenient online teaching and training services for students, teachers, enterprise mentors, outside experts, education management personnel and technical personnel, improves network delay and lag, improves communication and interaction experience of teaching and training users, promotes balanced development of education resources and promotes education equity. The four-dimensional virtual and real combined teaching scenario is shown in Figure 5.

RETRACTED

### 6.2. Design of Intelligent Teaching and Research Subsystem

The intelligent teaching and research subsystem consists of cloud listening and class evaluation and immersive online panoramic class tour function modules. Cloud listening and evaluating classes supports access to all classes anytime and anywhere, and real-time access to the listening and evaluating system for teachers' real-time picture acquisition, blackboard tracking and monitoring, student interaction and teachers' audio and video images under open classes, so as to carry out the listening and evaluating work for courses from a multi-dimensional and all-round perspective. Immersive online panoramic tour. To carry out online panoramic immersive tour, two modes are provided, one is automatic mode and the other is artificial mode. Automatic mode: including early warning mode and recommendation mode, through the AI algorithm of the system, combined with all kinds of teaching and management information to automatically analyze the class, the patrol staff can warn the problem class and recommend the quality class, the patrol staff can carry out targeted work, save a lot of manpower and material resources, improve the efficiency of the tour; Manual mode: Immersive panoramic tour is provided for the tour staff, which can fully realize the change of management concept from “blocking” to “estrangement” for the courses they are interested in, improve teaching level, standardize teaching behavior, and improve the quality of teaching and research. The smart teaching and research is shown in Figure 6.

### 6.3. Intelligent Teaching Management System Research

Intelligent teaching pipe system consists of five-dimensional open management of classroom and laboratory and equipment AI inspection function. Five-dimensional open management of classroom and laboratory, to create an open experimental carrier system with five dimensions of time, space, object, process and content, to realize unattended and automatic operation of carrier and equipment management, and to facilitate the promotion and operation of smart teaching and training platform. Intelligent device inspection provides automatic online inspection function for the central server, edge server and all kinds of terminal equipment (5G terminal, network terminal, breeding farm production terminal, etc.) of the intelligent teaching management platform, provides real-time warning and provides certain degree of self-operation and maintenance services.

RETRACTED

### 6.4. Intelligent Teaching Evaluation System Research

The intelligent evaluation subsystem carries out the teaching process evaluation and learning effect evaluation from the two dimensions of teachers and students, realizing the targeted online evaluation from the learning situation before, during and after class. The evaluation of smart is shown in Figure 7. The system supports a variety of evaluation systems, intelligent evaluation, real-time viewing of scores and effect analysis. Teaching process evaluation refers to the evaluation of the links or behaviors that affect the learning results of teachers in the process of teaching or interactive teaching. The assessment of teaching and learning effect, learning effect evaluation on learners learning after the completion of the final product testing or evaluation as overall rating of learners to participate in learning tasks, a full range of data, found that the participation of teaching and learning behavior model, the thinking process of digging their own to complete the task, real-time found problems in the process of problem solving, And then we can make immediate and accurate evaluation and intervention means through diversified and diverse forms. To evaluate the learning effect, students are evaluated comprehensively from the whole learning process, three-dimensional and multi-dimensional data concerns to diversified interactive forms, and guidance and intervention after evaluation are provided for them.

The intelligent teaching evaluation system is studied, which focuses on the two dimensions of teaching process and learning effect, obtains multi-dimensional teaching evaluation data from the intelligent teaching subsystem, establishes the intelligent teaching evaluation engine, and realizes real-time automatic evaluation feedback. The data of teaching content, teaching means, course explanation, teaching attitude, learning state, learning duration, learning concentration, homework, experiment and examination are obtained from the intelligent teaching subsystem. Data such as gender and professional title are divided into classification data, and data such as scores are divided into numerical data. The teaching content, teaching methods and other data were scored according to the degree of satisfaction and then converted into numerical data. The k-Centers clustering algorithm proposed by Gao Feng was used to analyze the teaching characteristics of animal husbandry, find out the commonness and differences, and provide useful guidance for teaching improvement in real time.

RETRACTED

The intelligent teaching evaluation system is studied, which focuses on the two dimensions of teaching process and learning effect, obtains multi-dimensional teaching evaluation data from the intelligent teaching subsystem, establishes the intelligent teaching evaluation engine, and realizes real-time automatic evaluation feedback. The data of teaching content, teaching means, course explanation, teaching attitude, learning state, learning duration, learning concentration, homework, experiment and examination are obtained from the intelligent teaching subsystem. Data such as gender and professional title are divided into classification data, and data such as scores are divided into numerical data. The teaching content, teaching methods and other data were scored according to the degree of satisfaction and then converted into numerical data. The detailed data planning is shown in Table 1. The k-Centers clustering algorithm proposed by Gao's was used to analyze the teaching characteristics of animal husbandry, find out the commonness and differences, and provide useful guidance for teaching improvement in real-time [21].

K-centers algorithm (hard partition and fuzzy partition), minimize the objective function as shown in formula.

(1) $$\begin{array}{c} F\left(W,Z\right)=\overset{k}{\underset{l=1}{\sum }}\overset{n}{\underset{i=1}{\sum }}w_{li}^{\alpha }d\left(x_{i},z_{l}\right)\text{.} \end{array}$$

The constraint conditions of fuzzy partition are shown in formula (2) and (3).

(2) $$\begin{array}{c} 0\leq w_{li}\leq 1,1\leq l\leq k,1\leq i\leq n, \end{array}$$

(3) $$\begin{array}{c} \overset{k}{\underset{l=1}{\sum }}w_{li}=1,1\leq i\leq n,0\leq \overset{n}{\underset{i=1}{\sum }}w_{li}\leq n,1\leq l\leq k\text{.} \end{array}$$

The constraint conditions of hard partition are shown in formula.

(4) $$\begin{array}{c} \min\;\left\{d\left(X_{i},Z_{l}\right)\right\}\leq \theta ,1\leq l\leq k\text{,} \end{array}$$

where, *α* ≥ 1 represents fuzziness, when *α*=1 is hard partition algorithm, and when *α*〉 When 1, it is fuzzy partition algorithm.

RETRACTED

The k-Centers algorithm process is described as follows:

1. Select the initial clustering center *Z*^(1)^ and the judgment *ξ* whether to terminate the iteration;
2. According to the initial clustering center *Z*^(1)^ , the membership matrix *F*(*W*, *Z*^(1)^) is obtained by minimizing *W*^(1)^. For *t*=1;
3. Minimize *F*(*W*^(*t*)^, *Z*) to obtain a new clustering center *Z*^(*t*+1)^. If |*F*(*W*^(*t*)^, *Z*^(*t*+1)^) − *F*(*W*^(*t*)^, *Z*^(*t*)^)|〈*ξ* is satisfied, stop.
4. Minimize *F*(*W*, *Z*^(*t*+1)^) to get a new membership matrix *W*^(*t*+1)^. Stop, if |*X* − *Y*|〈*ξ* is satisfied, Where *X*=*F*(*W*^(*t*+1)^, *Z*^(*t*+1)^), *Y*=*F*(*W*^(*t*)^, *Z*^(*t*+1)^); Otherwise, let *t*=(*t*+1) and return (3).

The complexity of the algorithm is O(n), and the computational complexity is approximately linear with the size of the data set, so that a large amount of data can be processed quickly and effectively [18], which meets the needs of real-time evaluation.

## 7. Conclusions

In view of the many challenges faced by agricultural and forestry colleges and universities in teaching, the intelligent teaching platform has been deeply studied, and the system architecture, application architecture and fusion network architecture have been proposed. Firstly, an in-depth study was carried out from the aspects of “openness, diversity, collaboration, equity and sustainability” of education, and it was proposed that online and offline teaching and double-teacher collaborative teaching should be carried out without being limited by time, space and safety prevention and control. Secondly, the teaching model of four dimensions from multimedia, real scene, virtual simulation to intelligent cultivation is studied. Thirdly, a smart teaching platform consisting of smart teaching, smart teaching research and smart evaluation is designed. The platform has been in operation for five years in relevant agricultural and forestry universities, which shows that the platform is reasonably designed, the sharing mechanism is complete, the cloud service is reliable, and it has the conditions for promotion and application in agricultural and forestry universities. However, the number of teaching resources related to real scene, virtual simulation and intelligent cultivation of the platform is limited, which is difficult to meet the teaching needs of all disciplines, and the corresponding new teaching resources are studied for different disciplines.

## Figures and Tables

**Figure 1:** Overall framework diagram of intelligent education platform.

RETRACTED

**Figure 2:** 5G converged network architecture diagram.

**Figure 3:** Intelligent education data center system cloud edge-end architecture diagram.

**Figure 4:** Architecture diagram of intelligent teaching resource sharing system.

**Figure 5:** Four-dimensional virtual and real combined teaching scenario.

**Figure 6:** Smart teaching and research.

**Figure 7:** Evaluation of smart.

**Table 1:** Teaching evaluation data set planning.

Dimension/Attribute	Type	Feature description
Teaching content, teaching methods, course explanation, teaching attitude, learning status, learning duration, learning concentration, homework, experiments to exams	Numeric	A 5-point scale is used. Note: The effect category is scored on a 5-point scale; numerical grades such as excellent, good, medium, pass and fail will be graded
Subject of the teacher	Can be classified	A total of 15 categories: Philosophy, economics, law, education, literature, history, science, engineering, agriculture, medicine, management, art, interdisciplinary, unknown
Professional title of teacher	Can be classified	There are four categories: Professor, associate professor, lecturer and assistant professor
Class student level	Can be classified	There are 2 categories: Undergraduate and graduate

## Data Availability

The data are available in the paper.
